# COVID-19: An Accelerator for Global Plastic Consumption and Its Implications

**DOI:** 10.1155/2022/1066350

**Published:** 2022-10-07

**Authors:** Moharana Choudhury, Subhrajeet Sahoo, Palas Samanta, Arushi Tiwari, Alavya Tiwari, Utkarsh Chadha, Preetam Bhardwaj, Abhishek Nalluri, Tolera Kuma Eticha, Arghya Chakravorty

**Affiliations:** ^1^Environmental Research and Management Division, Voice of Environment (VoE), Guwahati, 781034 Assam, India; ^2^Department of Environmental Science, Tezpur University, Tezpur, Assam, India; ^3^Centre for Life Sciences, Vidyasagar University, Midnapore 721102, India; ^4^Department of Environmental Science, Sukanta Mahavidyalaya, University of North Bengal, Dhupguri, West Bengal, India; ^5^Department of Chemistry, Indian Institute of Technology (IIT), Madras, Tamil Nadu, India; ^6^School of Chemical Engineering (SCHEME), Vellore Institute of Technology, Vellore, Tamil Nadu, India; ^7^School of Mechanical Engineering, Vellore Institute of Technology, Vellore, Tamil Nadu 632014, India; ^8^Department of Materials Science and Engineering, Faculty of Applied Sciences and Engineering, School of Graduate Studies, University of Toronto, Toronto, Ontario, Canada M5S 2Z9; ^9^Centre of Nanotechnology Research, Vellore Institute of Technology, Vellore 632014, India; ^10^Department of Materials Science and Engineering, Huazhong University of Science and Technology, Wuhan 430074, China; ^11^Department of Biology, College of Natural and Computational Sciences, Ambo University, Ambo, Ethiopia; ^12^School of Biosciences and Technology, Vellore Institute of Technology, Vellore, Tamil Nadu 632014, India; ^13^Research and Development Action Wing, Baranagar Baghajatin Social Welfare Organisation, Kolkata 700036, India

## Abstract

Plastic has been ingrained in our society. Repercussions on the usage of nonbiodegradable plastics and their problems have been recently realized. Despite its detrimental environmental impact, the COVID-19 epidemic has compelled worldwide citizens to increase their plastic use due to affordability and availability. The volume of hospital solid waste, particularly plastics, is overgrowing due to an unexpected increase in medical waste, culminating in the global waste management catastrophe. Henceforth, adopting good waste management practices along with appropriate technologies and viewing the current issue from a fresh perspective would be an opportunity in this current scenario. Accordingly, this review study will focus on the plastic waste scenario before and during the COVID-19 epidemic. This review also disseminates alternative disposal options and recommends practical solutions to lessen human reliance on traditional plastics. Further, the responsibilities of various legislative and regulatory authorities at the local, regional, and worldwide levels are addressed.

## 1. Introduction

Plastics are versatile, lightweight materials that can be processed using various manufacturing techniques with sizable market potential. It has been developed to overcome the shortcomings of materials found in nature. Plastics are polymeric chains consisting of monomers when joined in a repeating pattern, leading to the formation of plastics. Fossil sources are converted into these macromolecules through various methods, including polymerization, polycondensation, and polyaddition. Plastics can be classified into polymers of two categories: thermosets and thermoplastics. Polyethylene terephthalate (PET), polystyrene (PS), low-density polyethylene (LDPE), polypropylene (PE), high-density polyethylene (HDPE), expanded polystyrene (EPS), polycarbonate, polyvinyl chloride (PVC), polylactic acid (PLA), polypropylene (PP), polyethylene per (PHA), and polyhydroxyalkanoates are some of the most commonly used thermoplastics. It is possible to melt and process thermoplastics indefinitely without causing any chemical changes to the plastic material. It can sometimes be reshaped, reheated, and frozen without losing shape. At the same time, thermosets are types of plastic that undergo a synthetic irreversible transformation upon heating, resulting in a change in the structural orientation of the atoms. Once they have been warmed and shaped, these plastics cannot be resoftened or improved. Thermosets include phenolic resins, polyurethane (PUR), silicon, vinyl ester, acrylic resins, epoxy resins, and ureaformaldehyde (UF) resins. The inherent properties of plastic, such as low density, optical tunability, chemical inertness, reliability, durability, and ease of production [1, 2], have made it a viable alternative to traditional materials such as metal, ceramics, and wood.

According to the UN Environment Programme (UNEP), single-use plastics are any disposable plastic designed to be used just once, such as plastic bags. Single-use plastics are the most commonly used in packaging (approximately 50%), and this includes food packaging, bottles, grocery bags, containers, straws, cups, and cutlery, according to the Environmental Defence Fund [2]. Plastic drinking bottles, food wrappers, cigarette butts, plastic packs, stirrers, straws, and numerous forms of plastic bags and containers have all been designated as major environmental polluters by the UNEP [3]. Single-use plastics' most commonly used polymers include LDPE, HDPE, PET, PS, EPS, and PP. LDPE and HDPE are the most frequent polymers used for single-use plastics (Table 1).

Plastic bottles are purchased at around 1,000,000 per minute [3]. The consumption of plastic bags in the United States is estimated to be 4 trillion bags annually on average. In the most recent estimates, approximately one percent of plastic bags have been returned to the manufacturer for recycling [4]. A significant chunk of the 1,000,000 straws is consumed daily [5]. Straws are being phased out as a fashion accessory. Approximately 500 billion disposable cups are used yearly [6]. Despite their environmental benefits, single-use plastics are routinely thrown rather than recycled [7]. Compared to regularly putting one waste vehicle's worth of plastic (32 percent of the total 78 million tons) into the sea, what could be more damaging? By 2030, this rate is predicted to increase to two every minute; by 2050, it will reach four per minute [8]. More plastic will enter the oceans than fish in the coming decades.

Experts worldwide have come up with various measures for reducing plastic packaging use, including demands, roundabout fees, and even straight-up boycotting [9]. Plastic packaging bans are more prevalent in Africa and Asia, while Europeans are limited to just supporting the proposal. Although the research is inconsistent, it appears that a boycott or tax on plastic bags alters consumer behavior [10, 11], leads to a reduction in the use of plastic bags [12] along with an increase in the use of reusable bags [13]. However, while a ban on plastics has been linked to a reduction in plastic sacks in Portugal [14], its effectiveness in South Africa is limited [15]. Although Bangladesh and some regions of India have banned the use of plastic. These are ineffective and frequently disregarded in these countries [12, 16]. According to a recent report, south asian partners prefer to convert waste into usable energy over other methods of handling trash [17].

Mutha et al. [18] investigated the plastics material forecasts for India in 2006. They claim that between 2000 and 2030, total plastic consumption will increase by a factor of six, and that the calculated weighted average lifetime of plastic products will be nearly eight years. According to current reusing rates, the percentage of reusing is expected to decline from 47 percent to 35 percent by 2030. By 2030, total garbage accessible for removal (excluding reuse) is predicted to have increased by at least tenfold from its current level of 1.3 million tonnes. According to the findings, India needs a better waste management framework and administrative control from the government and industry [18]. Bhuyar et al. [19] investigated the ingestion of water bottles and plastic waste while traveling and the amount of plastic waste produced due to Nagpur railway station passengers' throwaway culture. According to the study, the average amount of plastic waste per person due to face mask use is 4 grams [20]. Unauthorized cloth pickers make a living by collecting low-value items from tracks and stages, such as drinking and soda pop jugs. The investigation concludes that a complete redesign of the waste management framework by rail route experts is required [19]. The ubiquitous existence of these elements worldwide demonstrates that they could considerably influence wildlife, ecosystems, the economy, and eventually, human health [21]. This study has highlighted the current state-of-the-art plastic waste before and during the COVID-19 epidemic and the current scenario (Table 2). Additionally, this review article will give a quick outline of the various strategies for managing plastic garbage.

## 2. Plastic Material Composition and Types

Most plastics contain binders, colors, plasticizers, fillers, and other additives. The binder determines the significant characteristics of plastic. Synthetic or natural binders may be used, such as casein, milk protein, or cellulose derivatives. However, synthetic resins make up the majority of the binders. It is also known as an ethylene polymer with the structural and empirical formulas, CH_2_ = CH_2_ and (–CH_2_–CH_2_–)_n_, respectively, synthesized at high temperatures and pressures to get desired products. Alkali, water, acids, and most organic solvents are all resistant to polyethylene [22]. The physical and chemical features of thermoplastics and thermosets distinguish them.

### 2.1. Thermoplastics

Thermoplastics can be melted, shaped, and resolidified using heat. They may be molded and hardened repeatedly. This attribute makes thermoplastic mechanically recyclable, an excellent feature to reduce waste. Thermoplastics are classified based on their structural organization, such as chemical bonding, as well as their level of characteristics and functionality. PET, or polyethylene terephthalate, is a form of thermoplastic that has been made from fossil fuels since 1940. PET has developed for industrial use, yet a substantial amount of it still finds up in the environment. According to a study published in 2016, the *Ideonella sakaiensis* bacteria can dissolve PET in order to use it as their only carbon source as well as degrade them into its precursors. This type of enzyme-assisted catabolic response makes them more bioavailable. Following this, several processes such as recycling, breakdown technologies, and bioremediation methods are used to treat plastic waste for the benefit of everyone involved, including the environment [22].

HDPE (high-density polyethylene) is an ethylene-based thermoplastic polymer. It is also known as polyethylene or alkaline. Polyethylene is created by polymerizing identical ethylene molecules. Polyethylene is a structurally ordered carbon and hydrogen-based unsaturated organic alkene. When compared to other thermoplastics, HDPE is a low-cost thermoplastic that has a linear structure and a minimal degree of branching. Low pressure (10–80 bar) and minimum (70–300°C) are used to create it and used for diverse applications [23]. Chlorine gas is most commonly used in the manufacturing of PVC. 16 million tonnes of chlorine are used in daily human activities (40% of annual production). Organochlorine produces the most PVC and is under regulatory and scientific attention because of its negative effects on human health. The majority of nonchlorinated plastic wastes have a greater negative impact on the environment than plastic garbage [24]. Vinyl synthesis, production of toxic compounds, and the excessive use of energy and resources at various stages of the manufacturing process collectively have severe environmental repercussions.

Both tubular methods and stirred autoclaving can be used to produce (low-density polyethylene) LDPE. LDPE has translucent and semirigid subunits (long chain), unlike HDPE, which is heavily branched with short- and long-chain monomers. To produce LDPE, free radical polymerization occurs at high temperatures and pressures (80–300°C). Short and long branches and subbranches of up to 40,000 carbon atoms can be found in this polymer. Tubular reactors are recently gaining higher importance than autoclaving because of their higher ethylene transformation rate [22, 24].

### 2.2. Thermosets

These are called as thermosetting or thermoset plastics. To create a three-dimensional link, polymers undergo heat treatments that result in a series of physical and chemical changes. Even though it is impossible to remelt or reassemble the thermoset molecules, at a physical state, they may be transformed into numerous materials with specific physical and chemical properties, as demonstrated by their ability to change from low viscosity liquids to solids that melt at a high temperature. Thermosets can be used in various ways; thanks to multiple additives that help them work better [22]. Low viscosity and a variety of additives allow thermosetting monomers to be utilized in diverse applications and make it easier for the user to change and customize the product. Organic monomers such as carbamate (urethane) are polymerized together to create polyurethanes. They have the same properties as thermoset polyurethanes, but they are easier to work with [25]. In addition to its adaptability, polyurethane's physical and chemical qualities allow it to be employed in various applications, such as in coatings, foams, and adhesives. Polyurethanes, like other polymers, utilize petrochemicals as a base or as a subingredient [26].

## 3. Plastic Waste Scenario before COVID-19

Plastics have taken on the role of modern workhorse materials in this era of modern technology. Since the 1950s, plastics manufacturing has been steadily growing due to an ever-growing human population [27]. According to the Plastics Europe Federation, more than 311 million tonnes of long-term degradability plastic were produced in 2014, up from 299 million tonnes in 2013 [28]. 85% of plastic is produced in the United States, Europe, and Asia, according to estimates. In the next 20 years, this figure will increase to 600 million tonnes [27]). According to Grand View Research, it is predicted that the global plastic market will develop at a compound annual growth rate (CAGR) of 3.2% from 2020 to 2027.

The plastic market is projected to grow due to increasing plastic use in a variety of industries such as healthcare and packaging. Packaging industries are the leading consumers of plastic, accounting for about 36.5% of the total usage [27], mainly due to its advantages like chemical/thermal resistance, high strength-to-weight ratio, and low cost. A wide range of materials, including containers and geomembranes benefit from these characteristics. PP, PE, PVC, PET, and PS are some of the widely manufactured plastics. PE and PET are two of the most common plastics found in the waste streams [27]. Polyethylene is available in a variety of densities, namely, exceptionally low density (XLDPE), low linear density (LLDPE), high density (HDPE), and low density (LDPE) [27]. As a result of their one-time use, plastic trash is generated. Large volumes of plastic garbage are generated every day as a result of human activities such as production and post-consumer scrap, which accounts for the majority of plastic waste [27].

The most frequent sort of plastic waste is thermoplastic, mainly postconsumer. The amount of solid plastic trash generated increases, but only a fraction of it is recycled. According to estimates, just 7% of the several tonnes of plastic garbage generated each year is recycled, 8% is burnt, and the rest is dumped [29]. Massive amounts of plastic waste have become a severe threat to the environment's long-term viability. Every year, around 300 million metric tonnes of plastic trash is generated [30]. At 42 million metric tonnes, or 13.1% of total waste, the United States produced the most plastic waste in 2016. In third place came India with 26 metric tonnes of solid trash, China with 22 million metric tonnes, and the EU-28 countries with 30 million metric tonnes of solid garbage, accounting for 11.7% of total solid waste [31]. When it comes to disposing of this garbage, the land is a significant consideration. So much plastic rubbish has been poured into the oceans that it has threatened the aquatic ecosystems' ecology, economy, and beauty [27, 29]. Almost 80% of the plastic waste found in the ocean comes from Asia [27, 32]. Plastic usage is undoubtedly harmful to both the people and the environment. Henceforth, many countries are minimizing plastic consumption by switching single-use plastics with paper-based packaging even before the COVID-19 outbreak.

## 4. Plastic Waste Scenario during the COVID-19

Plastic garbage generation has been made more difficult by the COVID-19 epidemic. PPE (personal protective equipment) items (including single-use plastics) and waste management practices that are harmful to the environment are not considered by this model (Figure 1). COVID-19's global spread has resulted in an increase in medical waste and single-use plastic waste. COVID-19 has accelerated plastic waste generation due to the inappropriate disposal of PPE. The amount of plastic wastes generated globally since COVID outbreak is presented in Table 3. Face masks and gloves were projected to decompose in less than a week [27, 33]. Single-use plastics have been a considerable advantage in the battle against COVID-19. Many countries have found that increased use of reusable shopping bags and coffee cups has reduced the virus transmission [27].

Countries with high COVID-19 cases are facing difficult time to manage the massive amount of hospital waste they generate. According to statistics gathered by Jordan's King Abdullah University Hospital, medical waste produced is ten times higher than before the pandemic. According to calculations, about 650 kg of medical waste is generated every day for 95 COVID-19 patients [27, 35]. Everyone, especially front-line employees and medical personnel, must wear adequate PPE because everyone requires personal protective equipment to avoid disease transmission. To safeguard people all around world, an estimated 65 billion gloves and 129 billion face masks would be required each month [27, 35]. Still, the indiscriminate use of PPE items by global citizens has become a concern due to poor product management and disposal.

Surgical masks and gloves should also not be used for 3–4 hours at a time. To avoid cross-contamination, the surgical mask should be replaced and thrown every 4 hours. According to Oceans Asia, masks may be spotted every 100 yards on Hong Kong's Soko Islands beach [27, 35]. Besides, pharmaceutical packaging waste is on the rise, as is the use of patient medications. Furthermore, the accumulation of plastic waste is aided by laboratory examinations, experiments, and blood tests. Because of the increased manufacturing and purchasing volume during this epidemic, the use of single-use plastics is expanding. Plastic demand for packaging is forecast to rise by 40%, while the market for other applications, such as medical applications, is likely to increase by 17% [27, 35]. Because everyone is concerned about their health and cleanliness at this time, most customers and providers will choose food wrapped in plastic containers or one time-use food packaging. Most restaurants replace used dishes and silverware. Supermarkets and food stores offer home delivery services to protect their customers' safety issues. According to a poll conducted in South Korea, the number of people purchasing food/groceries online has climbed by 92.5 and 44.5%, respectively, in the previous year [36]. In nations, such as Italy, Vietnam, and China, online purchases increased by 12–57% [36]. Profiting from this demand has resulted in an increase in the production of plastic waste including multilayered plastic, thin films, and foams. As the world prepared for the pandemic, the overuse of plastic resulted in a new scourge of plastic waste which we have been fighting at the expense of our ecosystem.

## 5. Global Threat

To match the amount of gasoline required to travel one mile, it takes around 14 plastic bags to make the trip. For the most part, plastic bags are only used for 12 minutes. It takes a long time for a plastic bag to disintegrate (at least 500 years) in a landfill. Unfortunately, the bags do not decompose in their whole. Instead, they have photodegraded, resulting in microplastics, which absorb toxins and damage the surrounding environment (Figure 2). According to Waste Management, every year, barely 1% of all plastic bags are returned for recycling. Despite the fact that the average family recycles only 15 bags each year, the rest winds up in landfills or the garbage. In the industrialized world, plastics are a by-product, and their global acceptance has expanded enormously in recent years, and it is likely to continue to do so in the future. The outcome was the development of organic polymers designed to alleviate the issues associated with traditional plastics [37].

Single-use plastic is extremely harmful to humans, animals, and aquatic life. Plastic particles are consumed alongside food by aquatic or marine oceanic creatures. Plastic cannot be processed, and as a result, it becomes lodged in their digestive system, causing severe medical problems. Poisonous synthetic compounds are released during the manufacture of single-use plastic sacks, which can cause serious illness in those who work with them. One of the major causes of natural contamination is plastic—individuals suffering from various diseases due to the contaminated environment. We must comprehend the issues that single-use plastic generates and eliminate its use. As a result, we must use less plastic unless necessary, shift to environmentally friendly products and services, and consider innovations that allow us to reuse plastics more effectively. To protect our planet, climate, and people, we must stop using single-use plastic. The Indian government has implemented a multiclerical strategy to reduce single-use plastics ‘use around the country in order to eliminate it from India by 2022. The cross-country ban on plastic items (such as plates, cups, bags, bottles, and straws) and other single-use plastics went into effect on October 2, 2019, intending to phase out single-use plastics from urban communities and towns that are most polluted. Given the foregoing, we owe it to ourselves, the earth, and all living creatures to cease using single-use plastic so that they might live healthy, happy, and prosperous lives. We produce massive amounts of single-use plastic regularly, the majority of which cannot be reused. Plastic sacks, polythene, plastic glass, straws, pop, water containers, and food bundling items are examples of single-use plastic. These single-use plastics are only used once before being discarded in the trash to be reused. Plastics, unlike natural materials, take decades to degrade completely. Plastic bags are nonbiodegradable and, in most cases, end up in a landfill, where they are covered, or in the water, where they eventually end up in the sea via various methods. They break down into minute particles in the soil and water bodies, but they do not disintegrate. They stay in dirt/water for over a century, delivering poisonous synthetic compounds and harming our lovely planet and climate in the process. In particular, plastic sacks that enter bodies of water are a major source of water contamination, and as a result, our current condition is deteriorating in every aspect [38, 39].

Single-use plastics are a clear indication of the problems that disposable culture brings along with it. Our reliance on them results in a tremendous amount of plastic waste generation amounting to around 300 million tonnes annually with more than half of it going into manufacturing single-use plastics which in turn cannot be recycled. Even though reusing as much plastic as possible lessens its impact on the environment, despite this, a whopping 91% of all plastic is never recycled again. In the absence of any other factors, it will eventually find its way into landfills or the environment. One of the most problematic aspects of reusing single-use plastic is that it falls into reusing hardware. As a result, reusing centers usually overlook single-use plastics, tiny things such as packs, straws, and flatware. Plastics do not degrade if left unattended; somewhat, they degrade by breaking up.

Plastics are gradually transformed into more modest pieces by the sun and warmth, eventually becoming microplastics. These small plastic parts, measuring 5 mm in length, are difficult to spot and are strewn. They end up in the water, where they are eaten by natural life, and then inside our bodies. Wildlife is particularly vulnerable to the dangers posed by microplastics because, when swallowed, they can quickly accumulate inside a creature's body, causing medical problems such as pierced organs and potentially fatal intestinal blockages. As a result, there is an increasing demand for low-cost biodegrdable materials to minimize emissions and address waste management challenges.

The employment of single-use plastic continues to be exceedingly ubiquitous in the daily lives of most American students despite a growing body of information proving its negative impacts on ecosystem, animal health, and human health. Although there are numerous low-cost alternatives, including metal straws, lunch boxes, reusable bags, and bottles, many communities still rely on the quick and cheap plastic choice. Bartolotta and Hardy [40] have suggested that the two most common reasons people will not choose a practical alternative are either they have forgotten their reusable goods at home or believe reusable items are unsanitary. Because the most common reason for not using a manageable thing fails to bring one, plastic alternatives are frequently available. Many people will conclude that using the more advantageous plastic option is not a big deal. This influence may be insignificant on an individual level, but it can have a significant cumulative effect if everyone adopts the same perspective. As a result of their routines, comfort, and general accessibility of single-use plastic objects, individuals find it impossible to change their behavior.

## 6. COVID-19 and Single-Use Plastics

It is believed to have originated from a creature and is causing significant respiratory problems in susceptible individuals [41] whereas the origins of virus are still unknown. On March 11, 2020, the World Health Organization's (WHO) Director-General proclaimed COVID-19 a pandemic, citing the transmission of 118,000 infected individuals to more than 114 nations [42, 43]. PPE became necessary to eliminate contamination among medical service employees treating symptomless and suggestive patients and allow public medical service frameworks to operate [44]. According to their estimates, medical service specialists require approximately 89 million clinical veils, 1.6 million goggles, and 76 million gloves every month [45].

Nonetheless, public worry about this highly contagious illness has accelerated the usage of personal protective equipment (PPE) by general public to limit the infection's unquantified spread worldwide. The projected monthly needs for personal protective equipment (PPE) at the time of deconfinement were around 1 billion face covers and 0.5 billion gloves [46]. According to WHO, the world's 7.8 billion individuals would use 129 billion face veils and 65 billion gloves each month if global comparisons were used [47]. The widespread and haphazard use of covers has caused controversy, with Western governments advocating against them because of lack of proof for assurance. A lack of proper handling, disposal and a misunderstanding that everything is alright could lead to an increase in dangerous activities [6]. A small group of researchers have been entrusted with reevaluating this choice with the hopes of reducing the spread of new coronavirus infections in the future [48].

It is extremely likely to have a significant impact on the plan to prevent another pandemic [49], and the researchers conclude that understanding HSW (hospital solid waste) disposal in isolated individuals with infectious diseases is critical. Although various researchers examined these strategies in an environmental setting, the following section will demonstrate the advantages of implementing these strategies to combat the COVID-19 virus without compromising public health. The hospital waste includes tissue waste, cytotoxic chemicals, and mixed garbage. In some cases, ignoring HSW can be dangerous [50]. Its distinguishing feature is that it may contain pathogenic agents that are hazardous to human health [51]. Approximately 15% of hospital garbage is deemed hazardous [52]. Human waste exposure causes the disposal of HSW [53, 54]. In Liberia, open during, indiscriminate dumping, and landfill account for roughly 10%, 65%, and 25% of solid waste disposal techniques, respectively [55]. Reliable waste management processes must include sorting, collection/transportation, storage, and disposal. [56, 57]. In the summer of 2012, some installations and hospitals used on-site waste management systems. As one of the critical components of the operation, effective use of protective equipment is required for waste management. Although some emerging economies have no plan in place to deal with the massive amounts of waste they generate [55], other countries have established policy frameworks. In the Nigerian town of Ogbomoso, there is no government-supported garbage collection, disposal, or recycling infrastructure in the local hospitals [58]. Incineration is a challenging method of waste disposal, but due to the high temperature, it would be highly effective on COVID-19 contaminated waste. Researchers found that pyrolysis and chemical disinfection are better alternatives to incineration and garbage disposal for managing medical waste [58]. The chemical disinfection of the ransomware virus is effective due to the sterilizing aspect, and the process is successful due to extremely high temperatures. For the management of HSW, these scenarios are advantageous. Comparable conclusions on the harmful effects of incineration and deposits compared to composting have been established based on a study for Gujranwala, Pakistan [59]. A viral transmission during COVID-19 can be successfully stopped if composting is adopted in separate vessel and proper waste handling techniques are used.

In addition, HSW can be self-sterilized, steamed, sterilized, and microsaved [60, 61]. These strategies are also effective against viruses. Other novel applications of low-temperature plasma, radiation, polymerization, and biological are converters can be considered. In areas lacking integrated waste management systems, infectious diseases are likely to spread quickly. Management systems for the use of HSW in hospitals are insufficient. In Aligarh, India, the Aligarh Institute of Medical Sciences faced a similar challenge [62]. The University Teaching Hospital of Lagos, Nigeria, also reported on the situation [56]. Iran's Hormozgan province was also plagued by problems [63]. Patiala City, India [64], Hormozgan City, Iran [63], and Anambra State, Nigeria all reported similar problems. There were also issues identified [65].

Despite the fact that the disease was unforeseen, current waste management failures in many developing countries have resulted in a revision of the existing waste disposal structure and system. In developing countries, government waste management is weak, inefficient, and unsustainable. New regulations developed and implemented across multiple governmental divisions rather result in a policy gap [66]. To prepare for the likely post-COVID-19 epidemic waste left behind by patients, a new long-term and sustainable policy is enquired to improve the current inefficient system. During and after the COVID-19 epidemic, the following sustainable methods for handling solid waste are recommended, including the use of PPE such as facemasks.

Waste management requires community participation from individuals. It is unsustainable to rely on the government to dispose garbage, especially given the inevitable increase in waste production, the anticipated future problem of more people, and the unforeseen pandemic COVID-19. By providing adequate equipment, scavengers and waste pickers will be protected from harm or disease, resulting in fewer workplace injuries. One of the most effective methods for preventing disease cross-contamination, such as the COVID-19 pandemic, is to incorporate source separation into the 3Rs of sustainable waste management (reduction, reuse, and recycling). To accomplish the United Nations Sustainable Development Goals (UNSDGs), source separation is required for healthy and livable cities and communities (SDG). Source separation is the best way to keep hazardous waste out of recycling or reusing recyclables to avoid health issues. For community waste treatment facilities, a set of regulations must be established. For biodegradable materials, waste disposal sites, and on-site waste processing facilities such as incinerators and autoclave machines must be available. Biodegradable incinerators are especially required on-site for waste treatment by communities and cities (Figure 3).

Decentralizing solid waste management (through multiple levels of management engagement) would ensure that various types of waste are treated appropriately and promptly rather than mingling or leaking into the environment. To solve hazardous waste problem, we can use a variety of procedures based on technical expertise, equipment availability, and financing capabilities, such as thermal treatment, microwave treatment, and so on [68, 69]. Still, the risk of COVID-19 snowballing due to improper EPI disposal cannot be overstated. In addition to the previously inadequate solid waste management system in developing countries, the significant increase in the number of cases necessitates practical actions to halt COVID-19 spread. Furthermore, the growing number of reports of COVID-19 infection in developing countries may aggravate the current strict rule, which requires facemasks as well as future lockout expansions in those countries, compounding the solid waste management challenge faced by used PPEs. Existing waste management policies in developing countries should be changed to address the environmental and health concerns of increased waste generation and unforeseen incidents like COVID-19 pandemic and others in a sustainable and effective manner. More importantly, COVID-19 solid waste pandemic requires sustainable solutions [67].

A novel approach developed recently is to determine which composts degrade biodegradable polymer-based biocomposites. Microbes naturally occur in compost, destroying biocomposites-based PLA (polylactic acid). Some modified biopolymers are recommended for environmentally friendly biocomposite biodegradable packaging. *Bacillus flexus* is also in charge of PLA-based microbiological data biodegradation. The inoculum is not required for the use of excellent and rich compost prior to biodegradation. Investigations in this field can help us understand how different bacterial strains react to thermophilic conditions when PLA-based composites are destroyed. The fact that the critical study only uses one compost type is a significant flaw. The microbial community's diversity has a distinct impact on all types of compost. They are also well suited for decomposition into biomedical biodegradable polymer biocomposite. According to research, the biocomposite of single-strain PLA has been successfully broken down by natural bacteria in composting settings. Microbial absorption and release from PLA matrix biofilters appear to have resulted in fractures and holes. The degradation/biodegradation of 90% of the carbon component in PLA composites takes about 180 days [70].

As long as the current epidemic persists, those who are unfamiliar with the management of solid hospital waste must be barred from handling it. If the government ignores the environmental impact of waste, it poses negative impact to ecosystem and public health; as a result, doctors must carefully manage medical waste disposal.

Specialized training for workers with few relevant skills is required for the management of infectious waste. If skilled labor is in short supply, workers must undergo training. Authorized parties should design and initiate advertisements for the general public. As a result, used gloves and covers would now be found as litter in public places, indicating that the general people's concerns regarding improper removal were not unfounded. Because it is primarily made up of plastics, this potentially enticing litter will survive in the environment, possibly dividing into microplastics, unless it is adequately gathered and disposed of face covers for single-use are typically composed of plastics like polyurethane, polyacrylonitrile, or polypropylene with orders based on filtration limits ranging from FFP1 (80 per cent) to FFP2 (94 per cent) and FFP3 (99 per cent) in European Union and from N95 (95 per cent) to N99 (99 per cent) and N100 (100 per cent) in the United States [71]. The recommended N95 veils, suitable for screening airborne particulates less than 0.3 microns in size by 95 percent, are made up of plastics like PP and PET, among other materials. Other disposable PPE items like cautious suits and veils, are primarily constructed of nonwoven fabrics commonly combined with PE, PP, and PET [72]. As a result, people inspired by the COVID-19 pandemic contribute to the growing plastic pollution problem by using and disposing of clinical waste. They can be transported all over the world [73], and under the influence of natural conditions, they can split into microplastics (tiny pieces of plastic that can be swallowed by animals or eaten by humans) [74, 75]. Because of long-term stability in environment, PPE deposits from COVID-19 phenomenon are likely to be a common rubbish ingredient in the background for a long time, with the potential to influence biota in a variety of ecological compartments and natural frameworks. During the epidemic, there may also be an accelerated demand for single-use plastic products as shoppers have shifted away from being concerned about environmental impact and toward using plastic packaging for reasons of hygiene and well-being [76]. Consequently, expanded interest for goods, medical services items, and internet business bundling are average, diminishing in the excess zones [77]. Thus, this pandemic altered utilization patterns by making money from the use of single-use plastic bundling, but it also caused a general decline in urban waste creation and hampered reuse efforts. However, the demand for disposable PPE in healthcare increased the design of clinical waste, sometimes beyond the therapy limit, necessitating the development of optional end-of-life medications.

Figures 4–6 clearly show the plastic production in various countries. The trends during COVID-19 in the selected regions where the consumption was reported were India, Europe, and China. India has shown an increase in the amount of produced plastics in 2020 during the COVID (Figure 4), which is evident that the services within the country may require a higher effort for controlling and recycling plastic waste. Whereas in Europe, the trends in plastic production remained stagnant during and before the COVID outbreak (Figure 6). European countries have a policy of recycling plastic waste on a large scale, which is only visible in upper-tier cities in India, which is also not completely followed. China reported an increment in plastic production in 2021 (Figure 5), but instead of 2020, there is an unusual trend where the plastic production since 2019, which decreased in 2020. The production remained within 10-11% from 2019 to 2021, which is not a major change on charts, but the values are very high.

## 7. Recommendations

Plastic utilization is unavoidable because of its lower price, flexibility, durability, suitability, and easy substitutability. They have a growing attraction among the people of all economic categories. Recovery, reuse, and recycling are possible to the maximum extent for plastic products of different kinds. On the other hand, plastic carry bags, including packaged plastics, are utilized without any control. Producers and consumers continuously invent new uses for carrying bags by giving up many natural products. So, the use of plastic carry bags expands at a faster rate. The used carry bags are carelessly discarded into the environment since they have no scope for recovery and resale opportunities. Discarded plastic bags create many problems for health, the environment, and resources. A total ban on carry bags of all kinds with the support of producers, consumers, and distributors within a specific period of time is the need of the hour. A practical, viable, flexible, and economically sound alternative for plastics in packaging will be a permanent solution to the problem. Plastic carry bags are invited danger, and they gradually entered into the consumption culture of developing countries from their developed counterparts who introduced them. But, developed countries with a solid institutional background are well-informed households backed by a good level of environmental education. Good economic environment, finding and following alternatives, and lesser disparities in many characteristics of the homes—reduce the use of carry bags, safely dispose/recover at the end in use stream, and recycle them appropriately. On this issue, developing countries lag in many respects. Above all, authorities need a strong political will to ban or control the packaged plastics and carry bags. Now it is time to join hands together and protect the environment from the mounting of plastic wastes, preserve land, water, and air, and make the world a better place to live. We could safely get relieved from the invited danger of plastics through a systematic and integrated management system.

India yearly produces nearly 9.4 million tonnes of plastic waste without any proper disposal system. Govt. of India implied a ban on single-use plastic items like straws, cups, spoons, bottles, and plastic bags from the second October 2019 on the 150th birth anniversary of Mahatma Gandhi. By the year 2022, the Hon'ble Prime Minister aims to abolish the utilization of single-use plastic entirely. To date, nearly sixty countries have banned using single-use plastic.

According to Deepak Ballani (DG, AIPMA) in a discussion in Rajya Sabha TV, “The problem is not with the plastic material but with the visible plastic pollution which starts from the littering habit of the society. As a material, plastic emits lesser greenhouse gas than bamboo, glass or even cardboards but its inadequate infrastructure to address scientific-based management of post-consumption waste to the segregation of its source, collection and disposal poses a problem. The people, the consumer, the municipal bodies are largely responsible for plastic waste management.” In the same discussion, Dr. Suneel Pandey (Senior Fellow and Director, TERI) said, “The thickness of plastic can be enhanced from 50 microns to 150 microns as it becomes more visible to the waste collectors. As well as Paper is not an alternative solution as using Paper leads to massive deforestation and Plastics evolved as an alternative of Paper previously to stop the deforestation.”

### 7.1. These Are Some Positive Approaches to Curb Single-Use Plastic Usage

Individual decisions and the aggregate movements they achieve—add up rapidly. They simplify only one trade, such as buying a water bottle that can reuse to save the climate and many plastic jugs every year. Here are a couple of more instructions for freeing your life (and your local area) of single-use plastics for good:

- Continuously gather a reusable sack when shopping (furthermore, yes—reusable sacks are preferred for the climate over plastics, late media asserts aside)
- Cook more frequently, to lessen your utilization of plastic-substantial take out compartments
- Purchase in mass. Keep away from separately bundled merchandise, similar to nibble packs
- What is the most sensible choice for reducing your impression and plastic waste? Online purchases, while sometimes less environmentally friendly than in-store shopping (avoid using the quick shipping option if at all possible), are nonetheless loaded with plastic when they get to their destination. Face-to-face purchases can be made via walking, bicycling, or taking public transportation
- Keep away from cling wrap through and through by putting away extras in reusable holders. Attempt reusable in addition to compostable wrap made using beeswax for an enlivening and straightforward alternative
- Purchase a bamboo or metal straw that is reusable. Pack it close by reusable cutlery (like bamboo, wood, or any metal chopsticks) for maintainable eating in a hurry
- Converse with the proprietors of the cafés you visit regularly. Please inquire whether they have nonplastic options in contrast to plastic straws, stirrers, or packs
- Stand up on the side of nearby plastic boycotts, regardless of whether by calling your nearby government agent, presenting an opinion piece to your city's paper, or essentially beginning discussions with neighbours
- Let organizations that make your significant items realize that you care about the bundling. Through social media call, or send letters to these organizations to request that they change to more substantial, recyclable, compostable, sustainable, and reused content bundling with less petroleum derivative inferred plastic

### 7.2. Few Recommendations during COVID-19 Pandemic

These workers which are prone to illness, collect garbage at dumps and further become contagious. Despite the fact that it is an effective way to preserve natural resources and avoid pollution, the existence of COVID-19 and the viruses globally spread means that the risk of infection must be reduced. Access to landfills and the availability of recyclables should be prioritized in efforts to protect these workers. Reduced recycling and increased use of single-use products should be encouraged for achieving SDGs (Figure 7).

Water treatment plants must increase their treatment efficiencies to prevent the novel coronavirus spread through the reuse of wastewater from entering the environment. This condition is necessary because incineration and deep burial are the only options available when dealing with human tissue in rural or isolated areas where a waste treatment facility is not readily accessible.

Face masks made of polymers are becoming increasingly popular, fuelled by environmental worries about plastic or microplastic contamination and waste management issues regarding waste management. It is recommended that biodegradable materials such as high molecular weight polyethylene (HMPE), artificial fibres, aramids, natural polymers, sponge nitrile, and polyurethane are utilized whenever possible in the construction of personal protective equipment. Manufacturing materials should also have a reduced carbon and water impact than materials that are chemically created.

### 7.3. Bioplastic—A Future Perspective

#### 7.3.1. EMBO

The company represents the bioplastics industry and promotes biodegradable and renewable bioplastics. According to the IUPAC, bioplastics are “biomass or plant origin monomers that can be designed at any point of development” [79]. Bioplastics are a type of modern plastic made from either recycled feedstocks or microorganisms. They are critical to a greener future because they drastically reduce environmental effects like greenhouse gas emissions and energy consumption. Bioplastic materials have now been proven to be a viable alternative to traditional plastics in several applications [80]. Bioplastics make up about 1% of the world's total plastic production, totaling 370 million tonnes [81]. Their annual growth rates, on the other hand, will be around 30% by 2025. Organic plastics can be entirely biodegradable for CO_2_ in months or years as part of the emerging circular biological economy. Rapid plastic waste processing is a significant factor in the international market for high-quality recycled plastics as part of the growing circular bioeconomy (e.g., absolute CO_2_ biodegradability without harmful products). Plants, microalgae, and cyanobacteria are used in solar-driven feedstock processing processes to create various biodegradable plastics and a long-term carbon sink infrastructure.

Food packaging, very light sachets, and farming applications have benefited from biodegradable plastic materials. For example, certified oil-biodegradable mulch films [82] have different environmental advantages depending on the application. Green polyethylene [PE] is different than traditional plastic in that it helps reduce greenhouse gas (GHG) emissions during the manufacturing process.

Biodegradable polymers are an additional benefit over nonbiodegradable polymers in that only a few biopolymers have outstanding mechanical qualities. Several materials, including starch, PVA, PLA, polybutyleneadipate (PBA), poly (PBA,” Butyleneadipates), and poly-3-hydroxybutyrate (PBA, PVA) [83, 84], have been used in the preparation of biodegradable packaging material. The relationship between biodegradation rate and mechanical qualities is inverse for the majority of packaging materials [85]. Biodegradability and high automation are two of PVA's advantages. It is also a thermally stable polymer with excellent chemical resistance, hydrophilicity, and high crystalline content [86, 87]. It is necessary to make modifications to improve the performance of the PVA packing film [88–90]. Most alteration techniques are employed to cross-link, categorize, and enhance mechanical, barrier, and thermal stability [91].

Green PE, derived during sugarcane processing, is the first certified renewable energy plastic globally, breaking new ground in the petrochemical industry as well as play a pivotal role in carbon capture and sequestration, contributing to climate change mitigation. Another effect of green plastic growth is the creation of SSCM (sustainable supply chain management). Supply chain management (SCM) is defined by flow, collaboration, stakeholders, relationships, value, effectiveness, and performance. SSCM combines economic, environmental, cultural, resiliency, and long-term objectives into business for sustainability [92, 93]. But green PE derivation from sugarcane processing is not sustainable because they compete for arable land, freshwater, and food production (Bastos2018), these are not fully agreed upon with the UNSDGs. Therefore, next-generation bioplastic manufacturing using microalgae can overcome these difficulties. It is also possible to employ saline or wastewater in microalgae systems, which may increase the likelihood of successful recycling by minimizing eutrophication and the need for stimulating chemical fertilizers in confined systems of nitrogen and phosphorus. Unlike fossil-based plastic, both natural and industrial composting environments can build biodegradability. Some biodegradable polymers such as polybutylene adipate and polycaprolactones are found in the fossil [94]. A scientist from Bangladesh recently invented a way of turning the fiber into cheap, biodegradable cellulose panels, converted into greener, plastically-like throw-away bags. These are plastic jute bags that are used for making burlap bags with plant fiber [95]. Although the Jute, known for its color and once-high pricing, is a “golden fiber,” its appearance has fallen as demand dropped. After three months in the soil, these bags are biodegradable and recyclable.

Compostable polymers are promoted as having environmental benefits [96], primarily when extracted from and regenerated by organic recycling, generated from renewable materials. Oil-derived plastics are altered by allowing the use of biodegradable plastics, which natural microorganisms can invest in the atmosphere or trash dumps [97, 98]. All plastics are, in general, nondegradable, but not all bioplastic is compostable. It is very crucial to understand the fact [99].

Pure nanocellulose produced by acid hydrolysis from agricultural waste material, such as jackfruit (*Artocarpus heterophyllus*), has recently been accepted by scientific community [100]. Several chemicals, including polyvinyl alcohol, glycerol, triethyl citrate, polyethylene glycol, and a unique filler (derived from *Boswellia serrata*, also named as frankincense,) were used for bioplastic formulation. A series of tests have confirmed the film's physical, electronic, thermal, and biodegradability. A different plasticizer was used during the film-forming to give the nanocellulose, plasticizer, and filler a more stable hydrogen bond [100]. This condition is because microalgae rapidly develop and do not compete with food stuffs [101]. Researchers have recently studied microalgae, the most common microorganism in seawater, and their potential as a renewable resource for bioplastics [102, 103]. Microalgae could be used as a direct source of biomass in bioplastics or extracted and processed into PHBs and starch, which can then be used in bioplastics. The algal-polymer blends are also created by extrusion, compression, heat molding, and other alternative techniques [104].

## 8. Conclusions

Reduced personal plastic usage is the most efficient method of reducing single-use plastic derived environmental pollution. Because of our current dependency on plastics, obtaining this perfect case scenario will be tough to accomplish [105–107]. People in developing and underdeveloped countries could benefit from being educated about plastics and implementing trash management strategies into their daily lives. Educating the public on negative adverse impacts of plastic trash on ecosystem and human health is essential to achieving this goal. If you compare the qualities of recycled plastic to those of virgin plastic, recycling is a time-consuming and expensive procedure with poorer properties [108–110]. The problems associated with the processing of plastic trash can be alleviated by technological innovation and the expediting of research and development efforts. One possible answer is the creation of biodegradable and environmentally friendly polymers. However, large-scale implementation and widespread adoption, on the other hand, entail a significant investment of time and resources.

## Figures and Tables

**Figure 1:** Circulation of microplastics in soil, water, and atmosphere [adapted with permission from [34]; Elsevier].

**Figure 2:** The interaction of microplastics with other environmental contaminants along with their influencing factors [adapted with permission from [34]; Elsevier].

**Figure 3:** COVID-19-related waste, and its potential long-term solutions [adapted with permission (under CC.BY. 4.0) from [67]; Springer].

**Figure 4:** Plastic production volume in India FY-2015-2021 https://www.statista.com/statistics/1067510/india-performance-plastics-production-volume/.

**Figure 5:** Plastic production volume in China FY-2012-2022 https://www.statista.com/statistics/1255628/plastic-product-production-in-china/.

**Figure 6:** Global plastic production volume FY-1950-2020 https://www.statista.com/statistics/282732/global-production-of-plastics-since-1950/.

**Figure 7:** Highlights for plastic product life cycle assessment and circular economy [adapted with permission (under CC.BY. 4.0) from [78]; MDPI].

**Table 1:** List of polymers used for the production of single-use plastics.

Types of Polymers	Applications
LDPE	Trays, containers, bags, food packaging film
HDPE	Freezer bags, milk/shampoo bottles, ice cream containers
PET (polyethylene terephthalate)	Various containers for water and other beverages, cleaning fluid dispensing containers, and biscuit trays are available
PS (polystyrene)	Cutlery, cups, and plates
EPS (expanded polystyrene)	Cups for tea and coffee, food packaging, and protective packaging for fragile objects are all examples of what we do
PP (polypropylene)	Microwave dishes, bottle caps, potato chip bags, and ice cream tubs

**Table 2:** “Reported COVID-19 cases, deaths, and estimated total plastic waste generation by region, measured in tonnes” [adapted with permission (under CC.BY. 4.0) from [20]; Elsevier].

Region	Population^a^	Total COVID-19 cases^b^	Total COVID-19 deatbs^b^	Facemask acceptance rate by population (%)^c^	Average facemask/capita/day	Estimated daily facemask disposed	Estimated plastic waste generated	Estimated plastic waste generated
							(tonnes)	per day (tonnes)
Africa	1,340,598,147	212,271	5,718	70	1	411,814,854	100,544,861	275,465
Asia	4,641,054,775	1,470,640	37,222	80	1	1,875,181,681	348,079,108	953,641
Europe	747,636,026	2,149,248	181,138	80	1	445,022,934	56,072,702	153,623
South America	653,952,454	1,267,858	54,648	75	1	380,414,703	49,046,434	134,373
North America	368,869,647	2,361,458	140,399	80	1	244,335,150	27,665,223	75,795
Oceania	42,677,813	8,896	124	75	1	21,682,379	3,200,836	8,769
Total						3,378,451,702	584,609,165	1,601,666

**Table 3:** Country-wise plastic consumption and wastage containment.

Year	Country	Statistics on plastic waste generation	Applied measures to contain the waste	Reference
2020	Worldwide scenario	As per the data released by World Health Organization (WHO), the requirement for medical masks, gloves, and goggles were around 89 million, 76 million, and 1.6 million per month during the pandemic.	Various countries came up with unique strategies to curb the growth of excessive plastic waste generation.	[1]

2020	China	The medical waste disposal on a national level as of January 2020 was 1164 t/d which gradually increased to 6066.8 t/d, which is an alarming rate.	With suitable technological advancement, municipal solid waste incineration facilities have been developed along with a robust epidemic prevention management system; the incinerated fly ash is managed as per the “Standard for Pollution Control on the Landfill Site of Municipal solid waste” (GB16889).	[2]

2020	Japan	Even before the pre-COVID-19 pandemic, Japan was dealing with issues like a trade ban on plastic waste from neighboring countries and population decline. As a result, waste management and treatment also became an unusual complication. During the COVID-19 pandemic, the demand for testing kits, disposable masks, etc., raised. As a result, the management of waste became even more complicated.	With the increase in several home deliveries during the lockdown, experts designed a prototype for a multibenefits mobility system that offers multiple benefits under one service. The benefits include transportation of goods and self-driving through either image recognition, GPS location information, or remote control. This prototype can also be considered a ‘moving trash bin.'	[3]

2021	India	Compared to the pre-COVID-19 situation, in India, the medical waste generated from hospitals, medical institutions, quarantine wards, and other departments was six times more, with more or less 517 tonnes of biomedical waste generated per day, including IV bags, surgical masks, and single use gloves.	For developing countries like India, solid waste can be conveniently handled through fundamental processes like incineration or landfilling. Plastic and healthcare wastes from medical institutions are pretreated through autoclaving and then conveniently disposed of in 1-2 meters deep burial pits in sanitary landfills.	[4]

## Data Availability

All the data are included in the manuscript.
